# Optimization: Molecular Communication Networks for Viral Disease Analysis Using Deep Leaning Autoencoder

**DOI:** 10.1155/2021/9949328

**Published:** 2021-12-13

**Authors:** A. R. Junejo, Mohammed K. A. Kaabar, Xiang Li

**Affiliations:** ^1^School of Control Science and Control Engineering, Harbin Institute of Technology, Harbin 150001, China; ^2^Gofa Camp, Near Gofa Industrial College and German Adebabay, Nifas Silk-Lafto, 26649 Addis Ababa, Ethiopia; ^3^Jabalia Camp, United Nations Relief and Works Agency (UNRWA) Palestinian Refugee Camp, Gaza Strip Jabalya, State of Palestine; ^4^Institute of Mathematical Sciences, Faculty of Science, University of Malaya, Kuala Lumpur 50603, Malaysia

## Abstract

Developing new treatments for emerging infectious diseases in infectious and noninfectious diseases has attracted a particular attention. The emergence of viral diseases is expected to accelerate; these data indicate the need for a proactive approach to develop widely active family specific and cross family therapies for future disease outbreaks. Viral disease such as pneumonia, severe acute respiratory syndrome type 2, HIV infection, and Hepatitis-C virus can cause directly and indirectly cardiovascular disease (CVD). Emphasis should be placed not only on the development of broad-spectrum molecules and antibodies but also on host factor therapy, including the reutilization of previously approved or developing drugs. Another new class of therapeutics with great antiviral therapeutic potential is molecular communication networks using deep learning autoencoder (DL-AEs). The use of DL-AEs for diagnosis and prognosis prediction of infectious and noninfectious diseases has attracted a particular attention. MCN is map to molecular signaling and communication that are found inside and outside the human body where the goal is to develop a new black box mechanism that can serve the future robust healthcare industry (HCI). MCN has the ability to characterize the signaling process between cells and infectious disease locations at various levels of the human body called point-to-point MCN through DL-AE and provide targeted drug delivery (TDD) environment. Through MCN, and DL-AE healthcare provider can remotely measure biological signals and control certain processes in the required organism for the maintenance of the patient's health state. We use biomicrodevices to promote the real-time monitoring of human health and storage of the gathered data in the cloud. In this paper, we use the DL-based AE approach to design and implement a new drug source and target for the MCN under white Gaussian noise. Simulation results show that transceiver executions for a given medium model that reduces the bit error rate which can be learned. Then, next development of molecular diagnosis such as heart sounds is classified. Furthermore, biohealth interface for the inside and outside human body mechanism is presented, comparative perspective with up-to-date current situation about MCN.

## 1. Introduction

In the last twenty years of 21^st^ century, coronavirus, alphavirus, fungal viruses, filamentous viruses, and members of the flavivirus family members cause more than 10 main viral diseases in the population. Significant overview of the 21^st^ century viral epidemics is presented. Timeline of 21^st^ century viral epidemics, from 2000 to the present day, is shown in Figure 1. Viral strains and the area of epidemics are indicated along with the timeline [1].

Over the past ten years, an interdisciplinary field of study called molecular communication networks (MCN) has been developed [2]. It bridges the areas of information engineering, and networking, and molecular biology [3]. The MCN focuses on realizing revolutionary new technology for a society that holds the promise for understated sensing and actuation capabilities inside the human body through a network of microsized devices [4]. These devices can use the existing natural signaling of cells, organs, tissues, and blood vessels to interact and communicate with the human body [5]. The MCN is moderately dissimilar from traditional electromagnetic communication in that MCN transfers information by using molecules for encoding, transmitting, and receiving information [6]. At present, scholars have contributed to MCN because of its potential to allow complex nanotechnology (NT) applications such as nanomedicine environment (NME) that requires microscopic entities to collaborate. For example, MCN can be used in in vivo biomedical applications [7], such as monitoring the healthcare industry (HCI) using biomicrosensors empowered by the *Internet of Biohealth things (IoHNT)* [8], target drug delivery (TDD), and so on. Presently, the most significant issue in the MCN is the way that the information is efficiently transmitted from one end transmitter (*T*_*x*_)  to another end receiver (*R*_*x*_) called the transceiver. The information is modulated by the physical properties of the molecules, where it is possible to change the type, volume, or time of releasing for the molecules to transfer the information. Each molecule diffuses in the medium after Brownian motion once emitted by the transmitter [9, 10]. During the transmission, due to the complex medium state, the signal suffers from interference and noise. MCN depends on the velocity of the fluid, the diffusion coefficient, the width of the bit pulse, and the response rate of the detector. The number of molecules consumed at each bit period is used at the receiver to demodulate the signals received. In MCN, modeling the entire system is optimized in a divide and conquer perception [11]. Commonly, the physical layer of the transmitter contains coding and modulation units, while the physical layer of the receiver contains equalization, demodulation, and decoding. Each component is individually optimized and requires a significant amount of expert knowledge. The enormous investigation has concentrated on optimizing each unit for various medium settings and demands for applications. The optimization of interaction subunits cannot assure global optimality for the entire interaction scenario [12]. In actuality, such execution is considered to be suboptimal [13]. In various composite MCN, it is challenging to directly find the transceiver design and medium model or other theories, which raises the difficulty of the study. Therefore, intelligent MCN is becoming an essential mainstream direction.

### 1.1. Role of Molecular Communications Networks (MCN) in Viral Disease Interaction

The related work based on the MCN is introduced inside and outside the body. The MCN gives us an exact representation of how the virus moves and distributes in the body over time. In the information environment, virus ions are considered information carriers, which transmit information (genome) from the transmitter location to the receptor which can be host cells in specific organs. The information transmitted by the virus is the function of the disease as shown in Table 1 [14]. A single virus ion is enough to enter the human body and cause viral illnesses as long as the host cell can attain virus binding. In addition to being disease-prone, vulnerable cells must also express receptors that bind to the virus and allow disease to develop, implying that they have the proteins and machinery required for virus replication

In MCN, micromachines are basic elements, and their sizes can vary from the micrometer level. These micrometers can carry drugs and provide therapeutic effects to humans during diseases. Drug-loaded micrometers are used for TDD. These drugs must act on cells because diseases are caused by cell disorders. To master the efficacy of therapeutic drugs, it must reach the target cells of the human body. In order to deliver the drug to the target in vivo, the drug-loaded nanomaterials must reach the nearby lesion cells and deliver the drug. In this work, we have studied all aspects of MCN and need a strong interaction mechanism, which brings many challenges. The first challenge is the effect of dynamic channel impulse response (CIR). During the interaction process, the molecules transported in the extracellular fluid move randomly according to Brown's motion. According to the Einstein diffusion theory, the CIR of the channel (medium) varies with time and the distance between the micrometers. We propose a different autoencoder (AEs), which sends a certain number of molecules to transmit bit 1 instead of sending molecules to send bit 0. On the nanoscale receiver, the signal is detected by sample, and the number of molecules is measured on each sample, and the concentration difference between two different samples is calculated. The transmitter sends signal molecules to interact with the receiver. These molecules reach the receiver, and the receiver detects the information in the molecule.

The transmitter and receiver are diffused mediums. For encoding and decoding, the difference between the samples of each interval is taken at the time *t*_1_ and, *t*_2_  so that the absolute difference between these samples is maximized. Then, the difference is compared with the threshold to make a decision that is advantageous to bit 1 orbit 0. When the bit 1 is received, the positive value of the concentration difference is given. When bit 0  is received, the negative value of the concentration difference is given. In MCN, bit 0 is represented by symbol [0, 1] and bit 1 is represented by symbol [1, 0]. Differential encoding and decoder *r* calculate the difference between peak values of received signals in continuous bit duration. When bit 0 is received, the difference is negative; when the bit 1 is received, the difference is positive. TDD is the most promising technology to deliver drugs to the target inside body. It can ensure that the amount of drug needed is intelligently located at a lower toxicity level. TDD can be achieved in two ways; first, nanoparticles carrying drug molecules are inserted through the cardiovascular disease and then reach the target MCN. Second, microdevices carrying drug molecules are implanted near target cells, bypassing the injection of cardiovascular disease [18].

### 1.2. Biohealth Interfaces for inside and outside Human Body MCN

The MCN mechanism provides a healthcare export that can use remotely measure biological signals and control certain processes in the organism required for the maintenance of the patient's health state. This technology can be further extended to use biomicrodevices to promote real-time monitoring of human health and storage of the gathered data in the cloud platform. This brings new challenges and opportunities for the development of biosensing networks, which will depend on the extension of the current inside and outside human body device functionalities. The improvement in the efficiency of HCI is expected, as these new devices will be able to interconnect among themselves and use the cloud to provide full-time access to all the data gathered by them [19]. To communicate with external networks, including the internet, these systems will require a translator device that will convert any molecular signal into electrical, which will continue to be applied for macrolevel computer networks, such as the Internet. The biointerface will also convert the different types of detected molecular signals to interface the exchange of information between the different micro networks placed inside the human body as shown in Figure 2.

Healthcare platforms, whole-cell biosensors are designed using synthetic biology (which is the formal method for the design of artificial systems using biological components) and can be applied to detect and treat CVD, assess the health risks associated with environmental pollution, and discover novel antibiotics, for example, cardiac pacing implant.

### 1.3. Cardiac Interfaces as Case Study

Inside the body, nanoscale devices have also been designed to interface the measurement of biochemical signals in the heart and circulatory system with external devices. For example, a cardiac interface was proposed to safely wirelessly power an implanted cardiac pacemaker (millimeter-scale device). The device is capable of closed-chest (rabbit) wireless control of the heart. The method allows to power nanoscale devices implanted with up to 5 cm  of depth. The powering device is placed outside the body, it has dimensions of 6  by 6 cm, and power the cardiac pacemaker using an electromagnetic signal with the frequency of 1.6 GHz. The device consists of a multiturn coil structure, rectifying circuits for AC/DC power conversion, a silicon-on-insulator integrated circuit (IC) for pulse control, and electrodes to stimulate the heart. Experiments were conducted with a cardiac pacemaker (2 mm  diameter and 3.5 mm of height) implanted into the lower epicardium of a rabbit, and its heart rate was monitored through an ECG. The size of the implant is 2 mm in diameter, 70 mg, and is capable of generating pulses at rates dependent on the extracted power. The device does not contain a battery; it is powered remotely. A portable, handheld power source was placed 4.5 cm distant from the device, after closing the chest, and it delivered 1 W of power to the cardiac pacemaker. The rabbit's cardiac rhythm was controlled wirelessly by adjusting the operating frequency. This powering system can be applied for any other optical or electrical stimulation task in the body, including neurons or muscle cells.

### 1.4. Deep Learning Techniques

The quick-growing deep learning (DL) has led to an innovative line of transmitter and receiver design. DL has been applied in various health care applications such as cancer diagnosis and prognosis prediction [20] (see also [21]). Current work displays that the transceiver can be jointly learned from data deprived of presenting any block-intelligent construction like modulator and channel encoder. This perception was first brought up in [22], in which an information system was deduced as an AE. However, DL could be applied in the interaction of physical layers and it is witnessed a dramatic performance improvement [17]. At present, DL clearly shows immense significance in breaking down the challenges of the information system. It is therefore inferred that DL boosts the output efficiency of each element in information networks or optimizes the full transceiver with an AE model [23]. The DL techniques allow the design of the MCN because of their abilities to approximate any nonlinear function. This motivates us to use the DL-AE to enable the transceiver to design the MCN. We proposed a model based on the multilayer perception deep neural network autoencoder (MLP-AE) and convolutional neural network autoencoder (CNN-AE), respectively, that can jointly optimize the transceiver design of the MCN system. A comparison between MLP-AE and CNN-AE is done in terms of SNR and BER. We have reported that under WGN noise, the proposed structure is capable of handling the challenge of mapping scenarios of various stages. Our techniques achieve efficient accuracy due to training epoch and less complexity concerning traditional model systems. By simulation, we compared SNR and BER and studied constellations from various AE configurations and prove that in a shorter training period, our suggested AE achieves a greater degree of reconstruction precision. We have illustrated the power of optimization approaches and the proper initialization of weight in providing ways to satisfy the demands of modern MCN applications for high-mobility and multienvironment applications.  Table 2 is a related work of MCN used by different techniques of DL.

The structure of the paper is organized as follows: Structure of the paper as in Section 2, we discuss the experimental design.  Section 3 gives results and discussion.  Section 4 summarizes our work in the conclusion.

## 2. Experimental Design

Autoencoder is used to optimize the design of the MCN transceiver as an end to end [32]. The goal of this section is to explain how to use MLP-AE and CNN-AE to design and optimize MCN. Then, we compare and analyze the performance of our techniques based on accuracy obtained after our AE has been trained and signal to noise ratio (SNR) vs. bit error rate (BER) for different configurations. In Figure 3(a) inside the body, the neuromuscular junction is one of the occurrences in biological communication systems where two cells communicate as a transceiver with each other using an intermediary molecule that propagates in the extracellular environment. When the muscle needs to be contracted, the nerve cell releases presynthesized special neurotransmitter molecules, called acetylcholine (ACh). These molecules propagate in this environment, and when they get close to the cell membrane of the muscle cell, they bond with the transmembrane receptors, called the ACh receptors (AChR). The neurotransmitters stay bounded for some time after which the bond degrades and the ACh molecules are again set free to the neuromuscular junction.  Figure 4(b) shows the MCN model using DL.

The transmitter selects the symbol *m* which contains *S*  bits of information, to be linked over a medium to the receiver. More clearly, the transmitter rule is to do a transformation to the symbol *m* so that Figure 3 produced transmitted signal *X* conquers *n* channel time slots. Then, a noisy version *Y* from *X* can be detected on the receiver side. Therefore, the receiver has to generate as similar as possible the approximation $\hat{m}\;$ of the initial symbol *m*. Hence, the system code rate is in equation (1).

(1) $$\begin{array}{c} \text{Code rate}=\frac{S}{n}\left(\frac{\text{bit}}{\text{medium}},\text{use}\right). \end{array}$$

### 2.1. Cumulative Density Function (CDF) Gaussian Model

The arrival of molecules in their nature is a binomial process. When considering multiple emissions, the number of molecules obtained is influenced by current and previous emissions over a period of time. It is expressed as a random binomial variable indicated as in equation (1). And *N*_*k*_^*T*^^*x*^ indicates the number of emitted molecules in the *k*^th^ symbol duration, *Pi* denotes the expected number of molecules absorbed by the receiver, while *β* (*n*; *p*) indicates the binomial distribution with *n* success and trail probability *p*. Because of the complexity of binomial random variables, the computational model is often approached by the Gaussian model [26] stated as in equation (3). The *N*_*i*_^*Rx*^ values are used to evaluate the cumulative density function (CDF) *F*_*Ni*_^*Rx*^(*x*) for Gaussian using the equation (4), where *p*(.) refers to the event probability. In our work, the additive white Gaussian noise (AWGN) is utilized. The noise proceeds digital values, though, its distribution role is estimated as in equation (5).

(2) $$\begin{array}{c} N_{i}^{Rx}∼\overset{i}{\underset{k=1}{\sum }}B\left(N_{i}^{Tx},P_{i-k+1}\right), \end{array}$$

(3) $$\begin{array}{c} N_{i}^{Rx}\sim ℵ\left(\overset{i}{\underset{k=1}{\sum }}N_{k}^{Tx}\;P_{i-k+1},\overset{i}{\underset{k=1}{\sum }}N_{k}^{Tx}P_{i-k+1}\;\left(1-P_{i-k+1}\right)\right), \end{array}$$

(4) $$\begin{array}{c} F_{N_{i}^{Rx}}\left(x\right)=P\left(N_{i}^{Rx}\leq x\right), \end{array}$$

(5) $$\begin{array}{c} \;N_{noise}\;\left(n\right)\sim ℵ\left(0,\sigma^{2}\right). \end{array}$$

### 2.2. MLP-AE-Based Model

As shown in Figure 5, MLP-AE is a feedforward neural network that maps the input to the output. An MLP-AE is consisting of neurons at multiple layers, containing the input (*m*), output ($\hat{m}$), and the number of hidden layers (*L*). Each layer in an MLP-AE has fully connected (FC) with the following layer, and each additional hidden layer needs an additional encoder and decoder. In the hidden layers, each neuron is activated with a nonlinear activation function. The idea is to train encoder (*E*) and decoder (*D*). Therefore, backpropagation using gradient descent [33] is appropriate for training an MLP-AE. In specific, AE learns a map from the input to itself through encoding and decoding stages. In specific, an MLP-AE can be regarded as an answer to equation (7) optimization problem. For MLP-AE, the *l* hidden unit activities, *h*_*l*_ is as in equation (8). Where *f* is the activation function (in this work, we use the softmax), *W*_*l*_ is a matrix of the parameter, and a vector of bias parameters bias_*l*_. Then, the *l* hidden layers output of the data is defined as in equation (9).

(6) $$\begin{array}{c} \hat{m}=D\left(E\left(m\right)\right), \end{array}$$

(7) $$\begin{array}{c} \;\frac{\min}{D,E}\left\|m-D\left(E\left(m\right)\right.\right\|, \end{array}$$

(8) $$\begin{array}{c} h_{l}=f\left(W_{l}h_{l-1}+{\text{bias}}_{l}\right), \end{array}$$

(9) $$\begin{array}{c} \hat{m}=f\left({\hat{W}}_{l}h_{l}+{\hat{\text{bias}}}_{l}\right), \end{array}$$

where ${\hat{W}}_{l}$ and ${\hat{\text{bias}}}_{l}$ is the decoding matrix and bias parameters, respectively.

### 2.3. CNN-AE-Based Model

Classically, a DL-AE can comprise a fully connected, layer, a densely connected layer, and a convolutional layer. FC or densely connected layers suffering from explosive dimensionality due to the tremendous number of connections between the neurons and therefore does not extend exceedingly to big-scale systems [34]. Besides, if the size of the system changes, the MLP-AE needs to be retrained since the number of tunable parameters differs mostly with the size of the system. To overcome these problems, we suggest an AE-based MLP comprising only convolutional neural network layers (CNNs). In a convolutional layer, each neuron will only be linked to a limited portion of the neurons throughout the preceding layer, and then all the neurons in the layer bear the typical set of biases and weights. This greatly lowers the overall amount of learning parameters. Our AE model-based learning essentially has two phases: (1) the encoder phase has sample input, convolution layers, and normalization layer and (2) the decoder stage includes feature coding input, deconvolution layers, and the reconstruction samples. The convolutional layers applied for both transmission and reception are a single-dimensional convolutional (Conv1D) layer. In our work, three layers were set up to be suitable to accomplish the finest possible bit error rate (BER) performance without losing any learning capability. From modulation perception, the Conv1D layers at the transmitter convert the input symbol sequence to a new signal illustration. The structure of the CNN-AE model is shown. We utilized ReLU as the activation function for the hidden layers in equation (11). For the output layer, we choose the softmax function as the activation function. We can describe the channel layer as the conditional probability density function *p* (*x* | *y*). Also, an additive Gaussian white noise with a fixed variance is added to the signals. Based on the system design of Figure 3, we propose a DL-assisted MCN transceiver, MLP-AE, and Figure 5, as CNN-AE, where the transceiver consists of DL-AE layers that are optimized jointly. The structure considered for MLP-AE and CNN-AE.

(10) $$\begin{array}{c} x=f\left(m\right), \end{array}$$

(11) $$\begin{array}{c} \text{ ReLU}\left(x\right)=\max\left(y,0\right), \end{array}$$

(12) $$\begin{array}{c} y=\text{softmax}\left(x\right)=\frac{\exp\left(X_{i}\right)}{\sum_{j}\exp\left(x_{j}\right)}. \end{array}$$

### 2.4. Implementation Details of MLP-AE and CNN-AE (Cardiac Interfaces as Case Study)

We design two AEs with identical configurations. Wach AE was trained on samples representing the recovered patients. We want to have the model with different parameters at the end of the training. To this end, we divide the samples to 10 groups of 20 samples {*gj*, *j* = 1, 2, ⋯, *n*} where *gj* is the *j*^th^ group of samples. To train the *i*^th^ model, *g*^*i*^ is set aside for validation and the nine remaining groups {*gj*, *j* ∈ {1, 2, .., *n*} − {*i*}} are used for training. Recall that each model is initialized with different parameters, trained on partially different training samples, and validated on the different validation sets. The 20 deceased samples are fed to each of the trained AEs. The samples undergo the compression and decompression routine of AEs. The decompression procedure is a loss so the reconstructed samples (after decompression) are not identical to the original ones. Moreover, the trained AEs exhibit different behaviors on the same input data since their parameters are different from each other. Therefore, feeding the same samples to the AEs will yield new samples which belong to the deceased class. The motivation behind the explained procedure is data augmentation to remedy the lack of enough samples for the deceased class. The reconstructed samples are attached to the original ones to yield a dataset of samples. A model was designed to classify samples as recovered or deceased. The model was trained using all samples. We apply 10-fold cross-validation during the training. Hence, the training sample size (samples of 9 folds) and the test sample size is 52 (samples of 1-fold). Using the trained one to classify the test data is shown in Figure 6.

## 3. Results and Performance Evaluation

The simulation findings are provided to illustrate the reliability of the suggested approach for various system settings. In this section, we compare the BER and SNR of the proposed CNN-AE and MLP-AE. The nonzero medium coefficients are believed to be drawn independently from a complex Gaussian distribution CN (0, 1). We, therefore, presume that the signals generated are similarly distributed. Besides, it is presumed that the noises from CN (0, *σ*) are drawn. This assumption enables a large range of SNR values to be identified by the proposed CNN-AE once it is well trained. In Figure 7(a), using MLP-AE techniques, BER is compared to CNN-AE data training at *K*_train_-20 and *k*_train_-100. It also indicates that our approach achieves a higher precision over the 100 training cycles. In Figure 7(b), using MLP-AE techniques accuracy is compared to CNN-AE data training at *K*_train_-20 and *k*_train_-100. The problem with improving the learning rate is that even after several iterations AE could not diverge, converge, or stop learning. If AE cannot converge, the end-to-end MC process can trigger bit reconstruction errors. By analyzing epoch and accuracy, epoch, and loss response, we can verify that AE is not convergent. Moreover, the slow rate of convergence is converted into higher BER and positioning in the AE-produced constellations. The proposed CNN-AE codec design can capture the MC medium/channel impairments by jointly optimizing transceiver operation. Through simulation, we compared *SNR and BER* and learned constellation from different MC medium configurations. Our results demonstrate that the optimization strategy and appropriate weights initialize the ability to provide new techniques for high mobility requirements. CNN-AE is described as a DNN model set, joint encoding at *Tx* corresponds to encoding, while joint decoding at receiver corresponds to the decoder. The reconstruction of information bits is optimized through the artificial neural network damage layer, which preliminarily verifies the good performance of AEs. An AE can learn without previous experience. Joint optimization entails pressuring the AE to obtain only the required features and characterize the data entered to store them in the block layer. After 100 epochs, all findings are acquired.  Figure 8 shows the rapid loss decrease in AE configuration. When we are talking about BER, the FNN-MLP has a low value of camper to all others. Finally, a comparison combination of both BER/SNR based on AE in Figure 8 is shown. In addition, Figure 9 shows a comparison of BER and accuracy performance between CNN-AE and MLP-AE with *K* = 20 and *K* = 100.

### 3.1. Comparison-Based CNN-AE and MLP-AE

The loss and accuracy plots of training the CNN on CT images are presented in Figure 7 showing loss and Figure 10 showing accuracy.

## 4. Conclusion and Future Work

Automated technologies for illness clinical diagnosis are increasingly desired as a result of viral disease analysis. DL-AE is a diagnostic and predictive tool for infectious diseases. The MCN mechanism maps to molecular signaling and communication found intrabody and interbody and characterized the signaling process between cells and infectious disease locations at various levels of the human body called point-to-point MCN. The DL-AE is a microscale system technology for TDD environments. Through MCN, a healthcare provider can remotely measure biological signals and control certain processes in the organism required for the maintenance of the patient's health state. This technology is further extended to use bionanodevices to promote real-time monitoring of human health and storage of the gathered data in the cloud. The performance has been evaluated in terms of BER and SNR. In this sense, it was emphasized that the accuracy rate of diagnosis can be improved via DL-AE by not needing any hybrid-complex models. The development of therapeutics/molecular diagnosis such as heart sounds was classified, when there is a problem with the heartbeat function, the heartbeat signal seems distorted. In future practices, advanced improvement learning techniques of our presented model should be used to disseminate a creative intellectual degree and improve convergence speed. We are optimistic that groundbreaking new research will emerge to aid in the fight against current and future pandemics.

## Figures and Tables

**Figure 1:** 21^st^ century viral disease epidemics.

**Figure 2:** The MCN that can be placed inside the human body and interconnected using biohealth interfaces. (a) Biohealth interface exchanges molecular data with the internet to enable the remote monitoring and control of intra-body devices. (b) An implanted nanopacemaker uses electromagnetic waves (EW) to stimulate the heart cells to exchange calcium ions.

**Figure 3:** The block diagram for the proposed MC transceiver design as MLP-AE.

**Figure 4:** (a) Inside the human body. (b) MCN model using DL.

**Figure 5:** The block diagram for proposed MC transceiver design as CNN-AE-AE.

**Figure 6:** The steps for implementing the proposed method.

**Figure 7:** CNN-AE and MPL-AE trained loss comparison.

**Figure 8:** Comparison of BER and SNR performances between the CNI- and MLP-based AE with *K* = 20 and 100, and Gaussian noise.

**Figure 9:** Comparison of (a) BER and (b) accuracy performances between CNN-AE and MLP-AE with *K* = 20 and 100.

**Figure 10:** CNN-AE and MPL-AE trained accuracy comparison.

**Table 1:** Related work of models for the viral air transmission medium.

Author	Propagation medium	Turbulence flow	Puff flow	Droplet evaporation	Droplet crystallization
I. F. Akyildiz et al. [11]	Air-based (transient air)	✓	✓	✓	✓
P. S. S. Tissera and S. Choe (2017) [15]	Air-based (cloud air)	✓	✓	✓	
K. Aghababaiyan et al. (2019) [16]	Molecular based (single droplet)	✓	✓	✓	
T. Nakano et al. (2012) [17]	Molecular based (particle dist.	✓	✓		
J. Ziv and M. Zakai (1973) [18]	Molecular based (concentration)	✓	✓		

**Table 2:** Related work of MCN used by different techniques of DL.

Author name	Year	Techniques used	Results
RF Mansour [24]	2021	DL-based variational autoencoder (UDL-VAE) model	Unsupervised deep learning-based variational autoencoder model diagnosis
Y Huang [25]	2020	CNN	Model-based detectors, data-driven detectors
TT Nguyen [26]	2019	AI	Artificial intelligence in the battle against viral disease
Qian [27]	2018	ANN	Prove that model-based and data-driven approaches generate the typical optimum receiver model, ensuring that the device model is correct
Alshammri [28]	2018	Joint ANN with the fuzzy method	Demodulate the data processed in the MCN system by on-off-keying modulation
Z. Qin [29]	2019	DL	DL enhances the intellectual communication of physical layers
He et al. [30, 31]	2019	DL	Model-driven DL decreases the demand for training data, results in faster deployment and reduces the risk of overfitting

## Data Availability

No data were used to support this study.
